The article "Cardiovascular events in early RA are a result of inflammatory burden and traditional risk factors: a five year prospective study" was published in 2011. Journal: Arthritis Res Ther.

# Cardiovascular events in early RA are a result of inflammatory burden and traditional risk factors: a five year prospective study

**DOI:** 10.1186/ar3442

**Published:** 2011-08-15

**Authors:** Lena Innala, Bozena Möller, Lotta Ljung, Staffan Magnusson, Torgny Smedby, Anna Södergren, Marie-Louise Öhman, Solbritt Rantapää-Dahlqvist, Solveig Wållberg-Jonsson

**Affiliations:** 1 Institution of Public Health and Clinical Medicine/Rheumatology, University Hospital, Umeå, 901 85, Sweden; 2 Department of Rheumatology, Sunderby Hospital, Luleå, 971 80, Sweden; 3 Department of Rheumatology, Sundsvall Hospital, Sundsvall, 851 86, Sweden; 4 Department of Rheumatology, Östersund Hospital, Kyrkgatan, Östersund, 831 83, Sweden; 5 Institution of Statistics, Umeå University, Umeå, 90187, Sweden

## Abstract

**Introduction:**

Co-morbidity and mortality due to cardiovascular disease (CVD) are increased in patients with rheumatoid arthritis (RA). Most published studies in this field are retrospective or cross sectional. We investigated the presence of traditional and disease related risk factors for CVD at the onset of RA and during the first five years following diagnosis. We also evaluated their potential for predicting a new cardiovascular event (CVE) during the five-year follow-up period and the modulatory effect of pharmacological treatment.

**Methods:**

All patients from the four northern-most counties of Sweden with early RA are, since December 1995, consecutively recruited at diagnosis (T0) into a large survey on the progress of the disease. Information regarding cardiovascular co-morbidity and related predictors was collected from clinical records and supplemented with questionnaires. By April 2008, 700 patients had been included of whom 442 patients had reached the five-year follow-up (T5).

**Results:**

Among the 442 patients who reached T5 during the follow-up period, treatment for hypertension increased from 24.5 to 37.4% (*P *< 0.001)), diagnosis of diabetes mellitus (DM) from 7.1 to 9.5% (*P *< 0.01) whilst smoking decreased from 29.8 to 22.4% (*P *< 0.001) and the BMI from 26.3 to 25.8 (*P *< 0.05), respectively. By T5, 48 patients had suffered a new CVE of which 12 were fatal. A total of 23 patients died during the follow-up period. Age at disease onset, male sex, a previous CVE, DM, treatment for hypertension, triglyceride level, cumulative disease activity (area under the curve (AUC) disease activity score (DAS28)), extra-articular disease, corticosteroid use, shorter duration of treatment with disease modifying anti-rheumatic drugs (DMARDs) and use of COX-2 inhibitors increased the hazard rate for a new CVE. A raised erythrocyte sedimentation rate (ESR) at inclusion and AUC DAS28 at six months increased the hazard rate of CVE independently whilst DMARD treatment was protective in multiple Cox extended models adjusted for sex and CV risk factors. The risk of a CVE due to inflammation was potentiated by traditional CV risk factors.

**Conclusions:**

The occurrence of new CV events in very early RA was explained by traditional CV risk factors and was potentiated by high disease activity. Treatment with DMARDs decreased the risk. The results may have implications for cardio-protective strategies in RA.

## Introduction

Mortality due to cardiovascular disease (CVD) is increased in patients with rheumatoid arthritis (RA) [1-8]. Several studies confirm that also cardiovascular (CV) morbidity is increased in patients with RA compared with controls [5,7-11]. According to most previous reports, traditional risk factors for CVD cannot fully explain this fact [3,5,10,12,13]. We have previously reported morbidity and case fatality due to myocardial infarction (MI) to be increased in patients with established RA from Northern Sweden, compared with the general population [9]. Hypertension was the only traditional CV risk factor that clearly predicted a CVE [9,13]. Although some controversy may exist over the statement [14], the inflammatory response is implicated as being predictive of CVD in patients with RA [13,15,16] and appears to potentiate the effect of traditional CV risk factors [17]. Most published studies in this field are, however, retrospective or cross sectional, and are often hospital-based and comprise information from medical records and various registers. Such studies are occasionally subject to deficiencies; for example, patients with low disease activity, patients moving out of the study region, and those suffering a premature death are lost. In order to focus on the progression of CVD during the course of a rheumatoid disease and to evaluate related risk factors in early RA, a prospective design is necessary.

The present observational study was designed to follow patients with early RA prospectively from disease onset. The aim was: first, to investigate the presence of traditional and disease related CV risk factors, at the onset of RA and during the first five years following diagnosis, in a large cohort of patients; second, to evaluate prospectively the predictive effect of these factors for CVD, as measured by the first CVE during follow-up; and finally, to assess the potential modulating effect(s) of the prescribed pharmacological treatment.

## Materials and methods

By reference to the nation-wide Swedish Rheumatoid Arthritis Registry [18] all eligible patients from the four northern-most counties of Sweden diagnosed with early RA (that is, symptomatic for <12 months), and fulfilling the American Rheumatism Association classification criteria [19] are since December 1995 consecutively included in a large survey on the progress of RA and development of co-morbidity, in particular CVD. By April 2008, 700 patients (481 women, 219 men) registered with newly diagnosed early RA had been included in the study at diagnosis of RA (baseline, T0). Of these, 442 patients reached T5, that is, they had suffered their disease for more than five years. All patients had been assessed regularly by their local rheumatologist during the follow-up period with special attention to established CV risk factors, any previous CVE, and clinical examination including blood pressure and laboratory tests. The following parameters were recorded at baseline and after 6, 12, 18, 24, 36, and 60 months: the 28-joint count of tender and swollen joints; a visual analogous scale (VAS) for pain and patient's global assessment; completion of a Health Assessment Questionnaire (HAQ) [20] and inflammatory markers, that is, erythrocyte sedimentation rate (ESR) and C-reactive protein (CRP). Disease activity score (DAS28) [21] was calculated. Lipid levels (total cholesterol (mmol/L), high-density lipoprotein (HDL, mmol/L) and triglycerides (mmol/L)) were analysed in the majority of cases at baseline, otherwise as soon as possible during the follow-up period. The presence of autoantibodies, that is, rheumatoid factor (RF), and anti-nuclear antibodies (ANA), was detected at baseline by the routine methods at each hospital. Antibodies against cyclic citrullinated peptides/proteins (ACPA) were analysed at baseline using enzyme-linked immunoassays (ELISA) for anti-CCP antibodies type 2. Genotyping for PTPN22 1858C/T polymorphisms was performed for the majority of the patients using the 5' -nuclease assay [22,23] and for HLA -DRB1 using polymerase chain reaction sequence-specific primers from a DR low-resolution kit and DRB1*04 sub-typing kit (Dynal, Oslo, Norway) as described previously [24]. In the present work the shared epitope (SE) alleles were defined as HLA-DRB1*0401 or DRB1*0404.

All patient records were carefully read and data collected according to a study protocol, both at inclusion at T0 and after five years at T5. In addition, the patients completed a self-reported questionnaire on co-morbidity at T0 and at T5 to further increase the validity of the collected data. Recorded variables were: all co-morbidity including previous CVE, that is, prior to inclusion, and new CVE during follow-up, that is, myocardial infarction (MI)/coronary artery bypass grafting (CABG), stroke/transient ischaemic attack (TIA)/deep vein thrombosis (DVT)/pulmonary embolism (PE), and ruptured aortic aneurysm. Myocardial infarction was recorded when the diagnosis had been made according to the World Health Organization (WHO) criteria [25]. A cerebrovascular lesion was recorded when intra-cerebral haemorrhage or cerebral infarction had been diagnosed by either computerized tomography or magnetic resonance imaging, or when a typical clinical profile of neurological deficits had persisted for more than 24 h. A TIA was recorded in cases when the focal neurological deficit of presumed ischaemic origin had persisted for less than 24 h. Deep vein thrombosis/pulmonary embolism was recorded when the diagnosis had been verified objectively (by phlebography, sonography, scintigraphy, and/or arteriography), or when the clinical signs combined with pulmonary radiography, electrocardiography, and laboratory changes resulted in full time warfarin treatment. The information regarding fatal cardiovascular events was obtained from the National Board of Health and Welfare. Furthermore, traditional CV risk factors (ongoing treatment for hypertension and current blood pressure, diabetes mellitus (DM), smoking (current and previous), body mass index (BMI)), rheumatoid nodules and time for development of extra-articular disease (EAD) [26] were registered. Cumulated pharmacological treatment was registered (months before inclusion and during follow-up) regarding corticosteroids and disease modifying anti-rheumatic drugs (DMARDs, that is, methotrexate, sulfasalazine, chloroquine, azathioprine, mycophenolatmophetil, myocrisine, auranofin, cyclosporine, leflunomid, alkylating cytotoxic agents) including biological agents (etanercept, adalimumab, infliximab, anakinra, rituximab) at inclusion and at follow-up. Treatment with non-steroidal anti-inflammatory drugs (NSAIDs), before inclusion (T0) and any period during the follow-up period (T5) was registered as "yes" or "no", as was treatment with statins - regarded as a proxy for presence of hyperlipidaemia. Time for treatment with selective cyclo-oxygenase-2 (COX-2) inhibitors was registered as exact as possible.

The first 128 patients included from two of the counties fulfilled the criteria for inclusion in the Swedish RA-registry but were, due to a lack of personnel resources, not recorded regularly. These patients were followed up in the same way as the other patients regarding base line data on inflammatory variables, autoantibodies, SE, pharmacological treatment, CV risk factors and previous and new CV events; however, they lack regularly recorded data on laboratory results, VAS scales and joint counts during the follow-up period. These patients did not differ significantly from the rest of the cohort when comparing ESR at baseline.

The regional Ethics Committee at the University Hospital of Umeå approved this study and all participants gave their written informed consent in accordance with the Declaration of Helsinki.

### Statistical analysis

The integral of disease activity, DAS28, was calculated in order to evaluate the total burden of disease activity over time and is referred to as the area under the curve (AUC) of DAS28 at 6, 12 and 24 months after inclusion into the study. When RA register data were missing, the last value was used to impute data once for each parameter assessed. Furthermore, for the regression analyses, imputations were made as follows: for AUC DAS28 at 6, 12 and 24 months respectively, the patient sample was divided into two groups, that is, censored and uncensored patients. Patients were censored after the time of the first event after inclusion or death or end of study. When values were missing for a single patient in each group respectively, data values were assigned by simple random sampling with replacement of values from patients with non-missing values, thus each missing value was replaced with an observed value. The same method was used for censored patients lacking data on levels of triglycerides.

For comparison of means of data and proportions between two sub-groups, unpaired t-test and Chi-squared tests were used, respectively. For comparison of recurrent data in the same individuals between variables at baseline (T0) and those collected at follow-up (T5), paired t-tests and McNemar's test for binary data were used.

For the regression analyses, time dependent variables were created for some variables: for extra articular disease (EAD), the variable time-EAD indicates when EAD occurred and time *t *when a CVE or a censoring has occurred. A dichotomous time-varying covariate was defined, with the value at time *t *= 1 if (*t *>time-EAD), otherwise this covariate was = 0. For treatment with corticosteroids and COX-2 inhibitors, dichotomous time-dependent variables were defined in a similar way. When defining the time-dependent variable for DMARDs, the accumulated number of months of DMARD treatment was also used; at each time *t *of an event and for every patient in the risk set, we determined the composition of the risk set and calculated the actual value of the variable DMARD at time *t *(DMARD(*t*)). For AUC DAS28, the time-dependent covariate AUC DAS28 was assumed to follow a step-function in which the values for AUC DAS6, AUC DAS12, and AUC DAS24 remained throughout the time intervals (0, 12), (12, 24) and (24, 60), respectively.

Cox proportional hazard simple regression models with fixed (time-independent) covariates were used to identify covariates associated with the first new CVE in the group of patients that were followed-up for five years following diagnosis (*n *= 442). For time dependent covariates, Cox extended models were also used with time-varying variables in simple regression models and in combined regression models with both fixed and time-dependent variables. Covariates reflecting disease activity, traditional risk factors for CVD and pharmacological treatment were considered in multiple regression modelling, based on clinical experience, previous studies and with statistical significance (*P *< 0.2) in simple Cox models, and tested in a few appropriate combined models.

All calculations were performed using PASW Statistics 18.0 (SPSS, Chicago, IL, USA).

## Results

In all, 700 early RA patients were attending the four rheumatology centres between December 1995 and April 2008. The first follow-up was in each case made five years after inclusion (T5); by April 2008, 442 patients had reached the five-year follow-up (T5). Twenty- three patients had died within the first five years following inclusion. All patients could be traced at the follow-up.

### Demographic data at T0 and T5 (Table 1)

**Table 1:** Demographic and clinical data in early RA at baseline (T0) and after five years (T5)

Variables	T0 (*n *= 700)	T5 (*n *= 442)
Sex, f/m	481/219	301/141
Age at onset of symptoms (years)	55.2 (14.3)	55.1 (14.2)
Duration of symptoms at inclusion (mo)	6.6 (3.3)	6.7 (3.2)
		
RF, n (%)	489 (76.4)	na
ANA, n (%)	130 (25.0)	na
Anti-CCP, n (%)	373 (67.8)	na
SE, n (%)	330 (56.9)	na
PTPN22 Tvariant, n (%)	167 (34.0)	na
		
ESR (mm)	31.5 (23.7)	20.0 (19.9)***
CRP (mg/l)	22.0 (24.6)	11.1 (14.3)***
DAS28^1^	4.8 (1.4)	3.2 (1.3)***
HAQ^1^	0.9 (0.6)	0.6 (0.52)***
Tender joints^1^	6.7 (5.8)	2.6 (3.7)***
Swollen joints^1^	7.4 (5.2)	3.2 (4.1)***
VAS pain (mm)^1^	44.5 (25.2)	28.7 (20.7)***
VAS global (mm) ^1^	45.3 (24.9)	29.8 (20.6)***
AUC DAS28 (6 mo)^1,^^2^	-	25.8 (7.1)
AUC DAS28 (12 mo)^1,^^2^	-	47.2 (13.5)
AUC DAS28 (24 mo)^1,^^2^	-	87.5 (26.0)
		
Extra-articular disease, n (%)^3^	-	21 (3.0)
Presence of nodules, n (%)	-	78 (20.7)

Mean (S.D.) or n (%).

*** *P *< 0.001, ** *P *< 0.01, paired t-test, for all patients who had reached the five-year follow-up, that is, who had data at both baseline (T0) and at follow-up (T5). NA, not analysed

^1 ^Regularly collected data from the RA-registry for 314 patients.

^2 ^AUC for DAS28 6, 12 and 24 months after inclusion.

^3 ^Criteria used for severe extra-articular manifestations: pericarditis, pleuritis, interstitial lung disease, Felty's syndrome, neuropathy, scleritis/episcleritis, glomerulonephritis, major cutaneous vasculitis and vasculitis involving other organs [26]. RA, rheumatoid arthritis; RF, rheumatoid factor; ANA, anti-nuclear antibodies; Anti-CCP, anti-cyclic citrullinated peptide/protein; SE, shared epitope; PTPN22, protein tyrosine phosphatise nonreceptor type 22; ESR, erythrocyte sedimentation rate; CRP, C-reactive protein; DAS28, disease activity score; HAQ, Health Assessment Questionnaire; VAS, visual analogous scale; AUC, area under the curve.

Descriptive data for all patients at baseline (T0) (*n *= 700) and for those having reached T5 (*n *= 442) are presented in Table 1. The mean age (standard deviation, SD) of the patient cohort at disease onset was 55.2 (14.3) years; for women this value was 53.7 (14.8) and for men 58.6 (12.6) years. The mean duration from the first signs of disease symptoms to inclusion at T0 was 6.6 (3.3) months, and was the same in both sexes. Regarding demographic data, the patient group that had reached T5 (*n *= 442) did not differ from the whole patient group (*n *= 700) at baseline. In the patient group that was followed up at T5 (*n *= 442), all of the variables reflecting disease activity (that is, ESR, CRP, DAS28) had decreased significantly (*P *< 0.001 for all three parameters) compared with baseline. The number of tender and swollen joints, HAQ, VAS pain and VAS global had also decreased significantly (*P *< 0.001 for all).

At the five-year follow-up (T5), 48 of the 442 patients (27 men, 21 women) (10.9%) had experienced a new CVE: 15 MI, 4 CABG, 23 stroke/TIA, 5 DVT/LE and 1 ruptured aortic aneurysm. Twelve of the events were fatal. In all, 23 of the 442 patients died from various causes during the follow-up period. Fifteen of the 48 patients who had experienced a new CVE had suffered an event prior to inclusion.

### Traditional CV risk factors at T0 and at T5

Data on traditional CV risk factors at baseline and after five years are shown in Table 2. In patients who had reached T5 (*n *= 442), treatment for hypertension had increased (*P *< 0.001) compared with T0, and both systolic and diastolic blood pressure had decreased significantly (*P *< 0.01 for both). The proportion of patients with type II diabetes had increased (*P *< 0.01). Significantly fewer patients were smokers (*P *< 0.001). BMI had also decreased significantly between T0 and T5 (*P *< 0.05).

**Table 2:** Cardiovascular risk factors and treatment in early RA at baseline (T0) and after five years (T5)

Variables	T0 (*n *= 700)	T5 (*n *= 442)
Hypertension, n (%)	170 (24.5)	164 (37.4)***
BP systolic, mmHg	144.1 (22.6)	141.2 (21.8)**
BP diastolic, mmHg	82.7 (10.3)	81.0 (9.6)**
Diabetes mellitus, n (%)	48 (7.1)	41 (9.5)**
BMI	26.3 (4.5)	25.8 (4.3)*
Smoking, present, n (%)	196 (29.8)	92 (22.4)***
Smoking, ever, n (%)	451 (69.5)	-
		
Previous CVE, n (%)	72 (10.4)	-
		
s-Cholesterol, mmol/L	5.6 (1.1)^1^	na
s-HDL, mmol/L	1.5 (0.5)^1^	na
s-Triglycerides, mmol/L	1.5 (0.7)^1^	na
Statin treatment, n (%)	54 (8.1)	71 (16.4)***
		
NSAIDs, n (%)	386 (58.5)	357 (82.4)***
COX-2 inhibitors, n (%)	82 (12.3)	112 (25.7)***
		
Corticosteroids, ever, n (%)	197 (29.1)	367 (72.7)***
Corticosteroids, months (T0 to T5)	-	22.3 (24.0)
		
DMARDs ≤3 months after inclusion, n (%)	-	393 (88.9)
DMARDs, ever, n (%)	-	429 (96.8)
DMARDs months (T0 to T5)	-	51 (16.4)
Methotrexate ever, n (%)	-	361 (81.5)
Biologicals, ever, n (%)	-	62 (14.2)

Mean (SD) or n (%).

*** *P *< 0.001, ** *P *< 0.01, * *P *< 0.05, paired t-test, for all patients who had reached the five-year follow-up, that is, who had data at both baseline (T0) and at follow-up (T5). na, not analysed

^1^analysed at baseline or as soon as possible during follow-up

BMI, Body mass index; BP, blood pressure; COX-2, cyclo-oxygenase-2; CVE, cardiovascular event; DMARDs, disease-modifying anti-rheumatic drugs; HDL, high-density lipoprotein; NSAIDs, non-steroidal anti-inflammatory drugs; RA, rheumatoid arthritis

### Pharmacological treatment at T0 and at T5

Data on pharmacological treatment are shown in Table 2. A total of 393 patients (88.9%) were prescribed DMARDs within three months following inclusion (T0) into the study. The mean time between the first symptoms of disease and DMARD treatment was 7.0 (0.3) months. During the first five years of disease, the patients had been treated with DMARDs for a mean duration of 51 (16.4) months. At T5, 429 (96.8%) of the patients were taking, or had been treated with, DMARDs for some time; 361 (81.5%) had received methotrexate, and 62 (14.2%) had been treated with biological agents.

### Predictors for a new CVE

In the evaluation of predictors of cardiovascular disease, simple Cox models revealed that an increase in the hazard rate of a new CVE during the follow-up period was predicted by higher cumulative disease activity (that is, both AUC of DAS28 at six months, and measured as a time dependent variable) and by progression of extra-articular disease, in addition to a greater age at disease onset, being male, having had a previous CVE and to traditional cardiovascular risk factors (diabetes mellitus, treated hypertension, higher triglyceride level).

Regarding pharmacological treatment, simple Cox models showed that a new CVE during follow-up was predicted by shorter duration of treatment with DMARDs during follow-up and treatment with corticosteroids both at/or before inclusion (T0) and during follow-up, before a new CVE. Also treatment with COX-2 inhibitors before CVE increased the risk in simple regression analysis. Treatment with DMARDs within three months of disease onset was protective, analogous to total treatment with DMARDs before a CVE (Table 3).

**Table 3:** Co-variates for a new cardiovascular event during five years after RA-onset in 442 patients.

Co-variates	HR	CI 95%	*P*-value
Sex f/m	0.314/f	0.177, 0.557	0.001
Age at onset of RA	1.060/yr	1.035, 1.086	<0.001
			
Diabetes mellitus	2.893/+	1.297, 6.452	<0.01
Hypertension, treated	4.066/+	2.308, 7.162	<0.001
BP, syst	1.015/mmHg	1.003, 1.026	<0.05
BP, diast	1.033/mmHg	1.003, 1.063	<0.05
S-HDL-chol	0.318/mmolL^-1^	0.090, 1.123	= 0.075
S-Triglycerides	1.919/mmolL^-1^	1.461, 2.521	<0.001
Statin treatment	2.237/+	0.950, 5.270	= 0.065
			
Previous CVE	5.912/+	3.210, 10.891	<0.001
			
AUC DAS28 (6 mo)	1.063	1.021, 1.106	<0.01
AUC DAS28^1^	1.025	1.010, 1.040	<0.01
			
Extra-articular disease^1^	3.343/+	1.421, 7.867	<0.01
			
Corticosteroids at/before inclusion	1.030/mo	1.004, 1.056	<0.05
Corticosteroids^1^	2.243/+	1.208, 4.164	<0.05
DMARDs within 3 mo^2^	0.402/+	0.200, 0.808	<0.05
DMARDs^1^	0.885/mo	0.200, 0.808	<0.001
COX-2-inhibitors^1^	2.392/+	1.206, 4.744	<0.05

Results of Simple Cox proportional hazards regression models, with fixed and time-dependent co-variates.

^1 ^= Time-dependent co-variate

^2^DMARD treatment started within three months from baseline (T0).

AUC, area under the curve; BP, blood pressure; CI, confidence interval; COX-2, cyclo-oxygenase-2; CVE, cardiovascular event; DAS28, disease activity score; DMARD, disease-modifying anti-rheumatic drug; HDL, high-density lipoprotein; HR, hazard ratio; RA, rheumatoid arthritis

The presence of ACPAs, RF, ANA, HLA-SE defined as *0404, *0401 in the present work, and PTPN22-T polymorphism had no statistically significant impact on the incidence of CVE.

When the impact of disease activity was evaluated in a multiple Cox model and adjusted for gender, hypertension and triglyceride level, a higher ESR at baseline independently increased the hazard rate of a new CVE. Treatment with DMARDs was protective, when included in the model above (Table 4). Adding age to the model resulted in a *P*-value = 0.19 for age. There were no significant interactions in the model. Figure 1 illustrates how the hazard ratio of a new CVE is potentiated by the combination of inflammatory activity (ESR) at baseline and cardiovascular risk factors (based on the variables in Table 4). The synergistic effect of increasing ESR at baseline and a higher triglyceride level is more than doubled by the impact of hypertension.

**Table 4:** Importance of potential risk factors for a new CVE in early- RA followed for five years.

Co-variates	HR	CI 95%	*P*-value
ESR, baseline	1.018/+	1.005, 1,030	<0.01
Triglycerides	1.853/mmolL^-1^	1.376, 2.496	<0.001
Hypertension	2.809/+	1.575, 5.008	<0.001
Female sex	0.449	0.249, 0.808	<0.01
DMARDs^1^	0.887/mo	0.856, 0.918	<0.001

Extended Cox multiple regression model, with fixed and time-dependent covariates.

^1^Time-dependent co-variate

Global Chi square (LR) = 131.45 on 5df (*P *< 0.001)

CI, confidence interval; DMARDs, disease-modifying anti-rheumatic drugs; ESR, erythrocyte sedimentation rate; HR, hazard ratio; RA, rheumatoid arthritis

**Figure 1:** **A new CVE is potentiated by the inflammatory activity and cardiovascular risk factors**. Estimated hazard ratio (HR) of a new cardiovascular event, (CVE), at a given time *t *during five years follow-up in patients with early rheumatoid arthritis (RA), taking inflammatory activity (erythrocyte sedimentation rate, ESR) at baseline (T0) and the level of triglycerides in consideration (median values as reference); **A**) without and **B**) with hypertension at baseline. The model also adjusts for gender and disease modifying antirheumatic (DMARD) treatment.

In a similar model, adjusted for gender, an increase in the incidence of CVE was indicated by cumulative disease activity (AUC DAS28) at six months (hazard ratio (HR) 1.064, confidence interval (CI) 1.027 to 1,102; *P *< 0.001) together with the presence of hypertension (HR 3.597, CI 2.028 to 6.380; *P *= 0.001), whereas DMARD treatment indicated a reduction (HR 0.891/month, CI 0.862 to 0.921; *P *< 0.001; data not shown).

With a focus on pharmacological treatment, DMARDs given before CVE decreased the incidence of CVE in the models presented. Treatment with COX-2 inhibitors before a CVE was a significant predictor of a new CVE in simple analysis. Adjusting for previous CVE did not change this relationship (HR 2.121, CI 1.072 to 4.2; *P *= 0.31). The impact of corticosteroid treatment could not predict a new CVE when adjusting the models for inflammatory activity including a model equivalent to table 4 (data not shown)

## Discussion

In patients with newly diagnosed RA followed for five years, a new CVE was predicted by high disease activity over time, extra-articular disease and by most of the traditional CV risk factors, that is, the presence of diabetes mellitus and/or hypertension at inclusion, and the level of triglycerides all predicted significantly a new CVE. Treatment with DMARDs decreased the risk whilst COX-2 inhibitors appeared to predict a new CVE.

We, and others, have previously shown that inflammatory activity is deleterious for the progression of CVD [13,15-17] although there are contradicting reports [14]. Most previous publications on CVD in RA are retrospective or cross-sectional and studies on inception cohorts are scarce. In one previous prospective study from disease onset, CRP at baseline was found to predict death due to CVD in a cohort comprising patients with polyarthritis rather than RA [27]. In patients with longstanding RA, CRP could also predict atherosclerosis, as measured by carotid intima media thickness, over an extended follow-up [28]. In the present study, ESR and CRP at inclusion did not predict future CVE in univariate analyses. However, when evaluated together with CV risk factors and DMARD treatment, ESR at baseline had an unfavourable prognostic significance for a new CVE. Furthermore, cumulative inflammation over time (that is, AUC of DAS28) could predict a new CVE in simple, as well as independently in multiple, regression analysis. Also, a more serious disease, as measured by development of extra-articular disease during follow-up, was associated with a new CVE consistent with previous reports on the predictive effect of extra-articular disease and RA-vasculitis [26]. Furthermore, an efficient suppression of disease activity, that is, treatment with DMARDS within three months following the onset of rheumatoid disease, significantly reduced the hazard of a new CVE as did more intensive DMARD treatment over time; the latter finding also applied to multiple regression models. It was also apparent that inflammatory activity is particularly dangerous in patients when combined with the presence of traditional CV risk factors such as hypertension and hyper-triglyceridaemia. These results emphasize previous findings by others [17].

Another finding of the present study was that treatment with COX-2 inhibitors was significantly predictive of a new CVE. Analogous with this, the consumption of COX-2 inhibitors was recently reported significantly more often in patients who developed an incident CVD in a three-year follow-up [29]. Treatment with COX-2 inhibitors during the first years after this study was initiated would preferably have been administered to patients with a known increased CVE risk to reduce the risk of complications such as gastrointestinal bleeding and water retention with concomitant CV complications. After rofecoxib was withdrawn in 2004, the opposite situation would be representative; that is, patients with an increased CV risk would not be treated with COX-2 inhibitors. After adjustment for a previous CVE, COX-2-inhibition was, however, still significantly predictive of a new CVE in our cohort.

Corticosteroid treatment appeared to be able to predict a new CVE according to univariate analyses. However, when the inflammatory activity was taken into account, corticosteroid treatment had no statistically significant impact on the hazard rate of CVE, implicating confounding by indication as an explanation for the results. Analogous to the findings presented, most longitudinal studies have not reported low-dose corticosteroid treatment to be a risk factor for CVD in patients with RA although this is still somewhat controversial [30]. We, and others, have reported a decreased risk for a new CVE following treatment with corticosteroids [13,16]. An attractive explanation would be that corticosteroid treatment reduces the deleterious disease activity by suppressing the inflammatory response. Although corticosteroids may have pro-atherogenic effects, as shown in patients with SLE [31], the net effect on CVD progression would be positive. A recent histological study of coronary artery tissue showed more unstable plaques in patients with RA compared with controls [32]. One possible pathogenic explanation to a favourable effect of treatment with corticosteroids would be a stabilization of such plaques.

We found that a new CVE was predicted by most of the traditional CV risk factors. This is at variance with most previous reports in which traditional risk factors have usually not been found to be of major importance for the development of CVD in patients with RA [5,10,12,13]. Hypertension increased the hazard ratio, both when measured by ongoing anti-hypertensive treatment and as raised current systolic and diastolic blood pressure. On this point, our data confirm previous retrospective studies [3,12,13,16,17,33] that have shown hypertension to be a significant predictor of a first CVE or death due to CVD. Over time, the treatment of hypertension had increased significantly at T5. In contrast, blood pressure at inclusion was higher than at the end of the follow-up period, probably reflecting the greater disease activity at disease onset, or as a result of anti-hypertensive treatment, and/or a better control of the blood pressure due to a stringent follow-up.

Diabetes mellitus was also significantly predictive of a new CVE. The influence of diabetes on future CVD has not been demonstrated in previous studies [5,10,12,13,16] although insulin resistance has been reported in RA patients [34,35]. In the QUEST-RA study, diabetes emerged as an independent risk factor in multivariate analyses but only for stroke [36].

Regarding hyperlipidaemia, statin treatment at inclusion (which can be considered a proxy for pre-existing hyperlipidaemia) increased the CV risk whilst a high HDL level decreased the hazard at statistical levels that were close to significance. In accordance with most previous studies, the level of total cholesterol was not predictive of CVD in this RA cohort. Dyslipidaemia, that is, a disturbed ratio of S-LDL/HDL cholesterol, may be relevant for the development of CVD in RA patients and appears to be dependent on higher disease activity [37-41]. In the present study, a higher triglyceride level increased the risk of CVE independent of sex, disease activity, anti-rheumatic treatment and hypertension. This is not consistent with previous studies [33,38,39,42]. In patients with SLE, hyper-triglyceridaemia is regularly reported as part of the lipid pattern commonly denoted as "lupus dyslipoproteinaemia" and comprises a decreased HDL level, an increased triglyceride level and no effect on the cholesterol level [43]. This pattern is, in SLE patients, associated with disease activity. One mechanism suggested to be responsible for this pattern is inhibition of lipoproteinlipase activity. In a previous study on patients with established RA, we found no increase in the level of triglycerides, but a relationship between lipoproteinlipase and inflammatory activity [44]. It is possible that the size of the patient cohort and the prospective design of this study is better equipped to reveal any important role for triglyceridaemia in atherogenesis in addition to RA. However, the level of LPL was not evaluated in this study.

The proportion of patients who smoked decreased over time. Smoking is a well-known risk factor for CVD morbidity and mortality in the general population, but was not a statistically significant independent predictor for a CVE in this prospective cohort of patients with RA. Only a few studies have reported an obvious negative impact of smoking on CVD in RA patients [12]. This is probably not due to smoking being less harmful in these patients but rather to its relatively small contribution to the total CV risk in patients affected with chronic inflammation [12].

Additionally, the mean BMI decreased significantly during the first five years of disease. Although most of the patients were adequately treated, with a mean DAS28 of 3.2 after five years, the decreased BMI may be a reflection of the continuing inflammation in RA leading to a certain degree of rheumatological cachexia [45]. In previous studies, a low, rather than a high, BMI has been associated with an increased risk of death due to CVD in patients with RA [46,47]. However, in these patients with early RA, the BMI did not show up as a significant predictor for a new CVE.

No association between the presence of RF or ACPA and future CVE was found. This is in contrast to a recent report [48] in which it was claimed that ischaemic heart disease is more frequent in RF- or ACPA-positive RA patients. However, the patient group in that study was hospital-based implying a more severe disease state than was present in our community based patient cohort. Furthermore, their cohort was not inceptional, with a mean disease duration over 10 years. The lack of association between PTPN22 polymorphism and future CVE was on the other hand in keeping with a recent study [49].

There are several strengths of the present study. First, the patient group comprises a large regional cohort and the prospective design involves few physicians at each rheumatology centre. In Sweden, essentially all patients with newly diagnosed RA are referred to a specialist. Thus, the results for the present cohort can be regarded to be general and, therefore, applicable to all patients with early RA. Furthermore, since only patients with very early disease were included, left censorship was avoided. Furthermore, repeated measurement of the parameters associated with inflammation made it possible to take variability in disease activity into account. Conversely, a limitation is the observational nature of this study with a risk of confounding by indication regarding the effects of pharmacological treatment. We tried to adjust for that by using multiple regression modelling in the statistical analyses when evaluating potential predictors of CVE. Another limitation is the relatively small number of events which restricts the estimation of possible multiple Cox models.

In the present prospective study evaluating risk factors for progression of CVE co-morbidity in patients with a recent onset of RA, we were able to show that the inflammatory status, both at disease onset and accumulated over time, was a strong predictor of a new CVE, with implications also for disease severity, measured as extra-articular disease. Furthermore, traditional risk factors and disease activity appeared to potentiate each other. Our data confirm the cardio-protective effect of disease modifying anti-rheumatic treatment. There were also implications of a harmful effect of Cox-2-inhibitions. Possibly due to the size and prospective design of this study, it was possible to show that most traditional risk factors for CVD are also of importance in early RA. In previous studies, their relative contribution to the total risk may have been concealed by the strong influence of inflammation. Because traditional CV risk factors are modifiable, a large effort should be made towards their prevention and treatment, in addition to the fundamental suppression of disease activity, when monitoring the care of patients with early RA. Our prospective data may add to the accumulated knowledge in future development of guidelines for the prevention of CVD in patients with rheumatic disease, work that is already ongoing in several countries and through international collaboration [50].

## Conclusions

In conclusion, we found that the progression of a new CVE in early RA was predicted by traditional CV risk factors, that is, the presence of diabetes mellitus and/or hypertension at inclusion, and the level of triglycerides, and was potentiated by high disease activity at inclusion and accumulated over time. Our data confirm the cardio-protective effect of disease modifying anti-rheumatic treatment. Given the current state of knowledge, it is important to suppress disease activity and great effort should be made to optimize the prevention and treatment of traditional CV risk factors in patients with RA.

## Abbreviations

ACPA: antibodies against cyclic citrullinated peptides/proteins; anti-CCP: anti-cyclic citrullinated peptid; ANA: anti-nuclear antibodies; AUC: area under the curve; BMI: body mass index; CABG: coronary artery bypass grafting; COX-2: cyclo-oxygenase-2; CRP: C-reactive protein; CV: cardiovascular; CVD: cardiovascular disease; CVE: cardiovascular event; DAS28: disease activity score; DM: diabetes mellitus; DMARD: disease-modifying anti-rheumatic drug; DVT: deep vein thrombosis; EAD: extra-articular disease; ELISA: enzyme-linked immunoassays; ESR: erythrocyte sedimentation rate; HAQ: Health Assessment Questionnaire; HDL: high-density lipoprotein; HLA: human leucocyte antigen; HR: hazard ratio; MI: myocardial infarction; NSAID: non-steroidal anti-inflammatory drugs; PE: pulmonary embolism; PTPN22: protein tyrosine phosphatise nonreceptor type 22; RA: rheumatoid arthritis; RF: rheumatoid factor; SE: shared epitope; TIA: transient ischaemic attack; VAS: visual analogous scale; WHO: World Health Organization.

## Competing interests

The authors declare that they have no competing interests.

## Authors' contributions

LI participated in the design of the study, collected and registered patient data, contributed to the statistical analysis and drafted the manuscript. AS, LL, BM, SM and TS participated in the collection and registration of the patient data. MLÖ performed the statistical analysis and contributed to discussions. SRD participated in the design of the study, collected patient data and contributed to a great extent to the discussion. SWJ was the principal investigator, designed the investigation, and participated in data collection, statistical analysis and drafting of the manuscript. All authors contributed to discussions and read and approved the final manuscript.
